The article "Development of University Music Education Based on Neural Network and the Reform of Music Education in Normal University under the Environment of Ability Education" was retracted in 2023. Reasons: unreliable results or conclusions; concerns about the data; concerns about the peer review; concerns about the citations.

# Development of University Music Education Based on Neural Network and the Reform of Music Education in Normal University under the Environment of Ability Education

**DOI:** 10.1155/2022/7605593

**Published:** 2022-09-23

**Authors:** Jinlai Dai

**Affiliations:** Xuzhou University of Technology, Xuzhou 221000, China

## Abstract

Competency education has grown in importance as a component of music education in teachers' colleges in the modern era. This essay conducts a thorough investigation into the evolution of college music education and the reform of music education at teachers' universities based on the notion of competency education. This essay highlights the crucial role that music education plays in competence education, with aesthetics at its center. It also examines the crucial part that music education plays in developing college students' all-round abilities. This study evaluates the reform process and current state of the music education curriculum system in teachers' universities based on these factors as well as the development trend of modern music curriculum reform, and it suggests various reform avenues. Additionally, a model for assessing the degree of music instruction is built in this research using the NN (Neural network) technique. This work employs MATLAB for empirical research in order to validate the validity of the method. According to experimental findings, this algorithm's evaluation accuracy can reach 96.11%, which is almost 13% greater than that of the conventional NN technique. The outcomes demonstrate the accuracy and dependability of this methodology. This study is intended to serve as a reference for the advancement of collegiate music education as well as the reform and innovation of music in teacher education programs.

## 1. Introduction

As an important part of competence education, music education in teachers' university is in the stage of continuous reform and improvement [1]. Music reform has also become an important and innovative content in education reform. At present, despite the rapid development of music education in universities, there are still outstanding problems [2]. There is a deviation in the orientation of the goal of music education in universities. The establishment of the goal of music education does not fully reflect the function of music education, which directly affects the effective implementation of music teaching. At the same time, the content of music teaching is single, the instructional facilities are imperfect, and the instructional purpose is unclear, which further hinders the rapid development of music education. Faced with the actual needs of basic music education today, especially the implementation of competence education, the diversity of professional skills and the comprehensive ability structure of quality cultivation of music majors in teachers' university have formed a great gap [3]. The synergetic theory of music education and competence education is to give full play to the unique aesthetic function of music education under the guidance of synergetic, so that it can coordinate, cooperate, infiltrate, and complement each other with each subsystem of competence education system, thus optimizing the overall function of competence education system [4]. Strengthening music competence education in universities is helpful to improve college students' aesthetic experience; it is helpful to stimulate college students' various perception and cognitive abilities; and it helps to cultivate students' rich imagination, expressiveness, and creativity, thus improving and perfecting their own comprehensive quality [5]. In light of this and the realities of universities, we should actively reform music education there; emphasize competency education to raise the general quality of students, and work to develop skilled music educators who can adapt to contemporary basic education. This dissertation presents a thorough analysis of the growth of college music education and the reform of music education in teachers' universities based on the notion of competency education.

Classroom quality assessment is an important link in instructional management. The content of instructional assessment in universities can be shown from the assessment index system [6]. It is helpful for school leaders and managers to understand the degree of realization of instructional objectives, and comprehensively and accurately grasp the situation of school teaching to improve the instructional level. Since the development of instructional assessment in universities, many universities have accepted the instructional assessment according to their own actual situation, and the instructional assessment in universities has also received extensive attention from everyone, which has aroused great attention from relevant social scholars. Teaching is a nonlinear classification problem, which brings great difficulties to comprehensive assessment [7]. With its unique properties of nonlinear processing, adaptive learning, and high fault tolerance, NN has been widely applied in many types of assessment problems. Additionally, NN offers special benefits in addressing the issue of assessing the instructional level [8]. Based on this, this study examines the fundamental theories and practices of conventional instructional assessment, as well as the characteristics and current issues with it. A prediction model based on BPNN (Back Propagation Neural Network) is suggested, and NN technology is brought into music instructional level evaluation on the basis of conventional instructional level assessment methodologies. This approach works well for predicting issues with unidentified rules. A collection of assessment index systems for the level of music instruction in universities are being built concurrently. The following are its primary research and work innovations:

1. This paper has some innovations in research ideas. The paper discusses the important position of music education with aesthetics as the core in competence education; at the same time, it studies the important role of music education in the cultivation of college students' comprehensive quality. Based on this, combined with the development trend of contemporary music curriculum reform, this paper analyzes the reform process and present situation of music education curriculum system in teachers' university, and puts forward some reform paths
2. There are some new research techniques in this paper: This study presents a hierarchical optimization of the instructional level assessment index system for the classroom. It is based on NN. It entails selecting topics for all-encompassing instructional level assessments as well as creating an index system for the assessments that is hierarchically optimized based on the faculties and universities that will be used. At the same time, a comprehensive fundamental data set of instructional assessment has been developed through the evaluation of instructional specialists, teachers' peers, and students

## 2. Related Work

Bonastre et al. took the “exploration of the nature of music education” as the breakthrough point to study the theoretical roots and value orientation of the nature of music education [9]. It re-examines music education and clarifies its positioning in the education system and in the all-round development of people. Tobias took “Music Education in the Quality Education System of Colleges and Universities” as the research theme, and provided a reference for the optimization and reform of music education in universities through in-depth exploration of the status, content, and methods of music education in college competence education [10]. Hayes introduced the necessity and background of music education and competence education in general universities [11]. The study points out that the goal of music education and the goal of competence education are consistent, which provides a necessary guarantee for the coordination of music education and competence education. Conway et al. analyzed the practice of basic music education [12]. It includes the empirical research of basic music education, the construction of basic music teachers, and the problems in the reform of basic music education; thus it clarifies the direction for the reform of the music education curriculum system in normal colleges and makes it more pertinent. Sims and Cassidy pointed out that because the time of vigorously practicing music competence education in universities is not long, there is still a lack of theoretical guidance in a certain sense; music education has not been effectively implemented, and there are still many problems that need to be solved urgently [13]. Daubney and Fautley believe that college students, as the main force of social construction in the new century, are the most valuable talents [14]. Therefore, improving the comprehensive quality of college students has become one of the main goals of talent training in universities. Gould et al. pointed out that at this stage, it is necessary to make it clear that music education is aesthetic education, and to deal with the relationship between academic teaching and quality training; the relationship between most students and the education of top students; and the relationship between students' active participation and teachers' leading role [15]. Lockhart et al. put forward reform suggestions for the problems in the current music curriculum system in teachers' university; at the same time, they clarified the guiding ideology that should be followed in the music curriculum reform in normal colleges [16]. Hessler et al. believe that through in-depth research, we should continuously improve various systems and give full play to the role of music education and instructional management model [17]. This is a major subject faced by music education in universities, and it is also a new field of theoretical research on instructional management. Amaele's research believes that the assessment of teaching work in universities is a scientific and reasonable judgment and measurement of the satisfaction degree of social values today; through instructional assessment, the future education work in universities can be better implemented [18].

This dissertation conducts a thorough investigation into the advancement of college music education and the reform of music education in teachers' universities based on the existing research and the concept of competency education. This study examines the reform process and current state of the music education curriculum system at teachers' universities in conjunction with the development trend of modern music curriculum reform, and suggests several reform avenues. The NN assessment model of college music instructional level assessment system is determined, including model design, network structure, learning parameters, and learning algorithm. It also proposes the design of hierarchical optimization of classroom instructional level assessment index system. The system utilizes object-oriented programming and B/S structure to achieve high levels of efficiency, networking, and intelligence in the assessment of instructional level.

## 3. Methodology

### 3.1. A Probe into the Development of Music Education from the Perspective of Competence Education

Art plays an irreplaceable special role in improving the overall quality of college students. Music education belongs to the category of art education and is one of the important ways to carry out art education in universities. Music is a kind of performing art, which expresses people's thoughts and feelings and reflects social real life through the artistic form formed by organized musical sounds. Music education is people-oriented and aesthetic-centered, which is one of the important means to implement aesthetic education and an important link to cultivate college students' comprehensive quality. From the level of music education in teachers' university, the connotation of competence education should include competence education such as artistic aesthetic quality, ideological and moral quality, cultural intelligence quality, and education and teaching. Its characteristics include comprehensiveness, development, and subjectivity. As an aesthetic education, music education should have a basic grasp of “aesthetic” characteristics. Aesthetics is a nonutilitarian or superutilitarian activity and experience, and its value lies in bringing people inner comprehension, satisfaction, and happiness. Aesthetic experience itself is the ultimate goal, not the end of acquiring other more important things. Music education in teachers' university should rationally adjust and structure the training of technical skills and rational quality. In this way, while imparting knowledge and skills, we can fully integrate the quality through the study of professional theory and academic theory.

Competence education has the following characteristics: (1) development and subjectivity: attach importance to human development and respect students' subjectivity; (2) internality: pay attention to the internalization mechanism in the process of education and teaching and emphasize the internalization of knowledge and educational influence into students' quality; (3) collectivity: competence education must face all students; (4) integrity: the implementation process of competence education must be to cultivate students' abilities in all aspects; and (5) effectiveness: quality-oriented education aims at comprehensively improving the basic quality and personality development of all students. Quality-oriented education points out the development direction and provides a rare opportunity for the reform of music education in teachers' university. At the same time, music education is an important part of competence education, and it is of great significance to further promote competence education by strengthening the reform of music education in teachers' university. As the implementation of competence education, music competence education is an important content to achieve the goal of cultivating all-round development talents. It can not only cultivate students' ability to feel, appreciate, express, and create beauty; moreover, music aesthetic activities can enlighten students' wisdom, develop students' potential, promote the harmonious development of personality, and have an important impact on people's ideological and moral concepts and intelligence It can be said that music education is fundamentally aesthetic education, rather than the education of pure knowledge and skills. The whole process of music education should be embodied in the process of educating people with aesthetics as the core. Music teaching can cultivate students' temperament, cultivate noble sentiments, construct a full inner world, and promote students' intellectual development through aesthetic links; Enhance creativity to achieve the educational goal of improving students' overall quality and making students' body and mind develop harmoniously.

Music education is open, and it can flexibly incorporate aesthetic activities such as music inside and outside the school into daily teaching. For example, organizing concerts and communicating with off-campus art groups can effectively promote college students' appreciation level, communication ability, sense of cooperation, and collectivism. Although musical language cannot express systematic thoughts and theories, it shows a certain realm and charm, which is not only easy to directly penetrate into college students' feelings, affect their spirits and cultivate their sentiments but also it is easier to guide college students to establish correct moral outlook, outlook on life, and values. Music education is a basic education with students as the object, music art as the carrier and aesthetic education as the core. Its fundamental purpose is to cultivate all-round development. Therefore, in music education in universities, we must always set up the concept of “student-oriented” education and teaching. At present, the establishment of training courses for music majors in teachers' university cannot still follow the past one, which only focuses on the simple introduction of famous works in the history of Chinese and foreign music, as well as the technical graphical music appreciation. It must organically introduce and integrate many disciplines in musicology, such as music history, music and performance, music and national culture, music aesthetics, and aesthetic psychology. In the process of music education, when college students are immersed in the feeling and appreciation of beauty, and are nourished and coordinated by beauty in spirit, they can make agitation tend to be peaceful, tension tend to be relaxed, and sadness be soothed through artistic sound waves, rhythm changes, and speed to adjust their psychological balance. This is conducive to the healthy and harmonious development of body and mind. As music education in universities from the perspective of competence education, the correct establishment of goals is directly related to every link of music education practice, such as curriculum setting, instructional methods, and compilation of instructional materials. In the curriculum structure of music major, quoting some knowledge systems of literature and art will surely help music major students in teachers' university to improve their music appreciation ability. Create a more comprehensive person with sound development in both perceptual and rational aspects. It opens up a new way for music education in teachers' university, in which three qualities, namely professional quality, thinking ability, and humanistic spirit, are isomorphic and symbiotic. We must constantly think about creating a new mode of college students' music education, earnestly strengthen college students' music education, and improve their comprehensive quality through the improvement of college students' music education.

### 3.2. Design and Implementation of Instructional Level Assessment Model Based on NN

NN technology [19, 20] is a new technology with development potential. It can use its own nonlinear ability to process related information. Neuron is the most basic unit component of NN. It is the basic processing unit of neuron NN, which is generally a nonlinear device with multiple inputs and single outputs. When a large number of neurons form a network, it will have a good function of processing and storing various types of information, and can complete difficult calculations. The action of neuron is very simple. It only multiplies the input vector by the weight vector, and then gets the output value after a transformation. As the basic unit of NN, neuron model has three basic elements: (1) a group of connection weights; (2) a summation unit; and (3) a nonlinear excitation function.  Figure 1 shows the neuron model.

The forward propagation of information and the backward propagation of mistakes make up BPNN. Error back propagation begins when the actual output differs from the anticipated result. This NN-like model is a multilayer mapping NN that employs the lowest mean square error learning strategy. It is currently one of the most popular NN models. The repetitive process of information forward propagation and error backward propagation involves NN learning and training as well as constant weight adjustments at all levels. The nonlinear classification may be achieved and any nonlinear function can be approximated with any accuracy by modifying the link weights in BPNN and the network scale. Error correction is the most fundamental BP algorithm principle. In order to reduce the error, the gradient descent approach is utilized to alter and update the connection weight of the network through the back propagation of the network output error.

The establishment of a scientific and systematic instructional assessment system can enable teachers to grasp the problems in their own instructional process at the first time, and make adjustments as soon as possible, to make it more in line with students' learning habits or interests, thus improving the instructional level [21]. Judging from the existing assessment system of instructional level, the design of indicators is concentrated in the following aspects: (1) instructional attitude; (2) instructional content; (3) instructional ability; (4) instructional methods; (5) instructional and educating people: and (6) instructional effect. The traditional instructional level assessment system makes it difficult to reflect the principles of comprehensiveness, authenticity, scientificity, objectivity, and democracy. Therefore, the first premise of constructing the instructional level assessment system in universities is to define the subject and object of instructional level assessment in an all-round way. Combining with the actual instructional activities and referring to the assessment index system of instructional level in universities; this paper constructs the assessment index system of music instructional level. When designing the assessment index system of music instructional level, this paper tries to embody the principles of scientificity, comprehensiveness, accuracy, and measurable operability. The specific content of the assessment index system of music quality is shown in Table 1.

All-round classroom instructional level assessment system includes teacher's instructional assessment system and student's learning assessment system. Each assessment system includes different assessment index systems, which are independent and interrelated. On this basis, after sorting out the initial data, qualitative and quantitative analysis, the proportion of assessment indexes in the whole index system is preliminarily formed.  Figure 2 shows the structure of BPNN model.

Step function is another name for threshold function. When the activation function is simply used to assess if the network input received by neurons exceeds the threshold, this function is employed instead. The equation reads as follows:

(1) $$\begin{array}{c} f\left(x\right)=\left\{\begin{array}{cc} 1 & x\geq 0,\\ 0 & x<0. \end{array}\right. \end{array}$$

The most fundamental activation function is linear function. It contributes to the appropriate linear amplification of the network input that neurons receive. Its basic format is

(2) $$\begin{array}{c} f\left(x\right)=kx. \end{array}$$

Among them, *k* is the amplification factor; *c* is the displacement. They are all constants.

The linear function is very simple, but its linearity greatly reduces the performance of the network, and it even degenerates the functions of multilevel networks into those of single-level networks. Therefore, it is necessary to introduce nonlinear activation function into NN:

(3) $$\begin{array}{c} f\left(x\right)=\left\{\begin{array}{cc} 1 & x\geq x_{0},\\ ax+b & x_{1}\leq x\leq x_{0},\\ 0 & x\leq x_{0}. \end{array}\right. \end{array}$$

In this paper, the activation function of each layer of the network is a unipolar S-shaped function, namely,

(4) $$\begin{array}{c} f\left(net\right)=\frac{1}{1+e^{-net}}. \end{array}$$

Implicit layer adopts formula is as follows:

(5) $$\begin{array}{c} H=\sqrt{N+M}+\alpha 0<\alpha <10. \end{array}$$

Among them, *H* is the number of hidden layer nodes; *N* is the number of input layer nodes; and *M* is the number of output layer nodes. The weight adjustment amount for each network layer may thus be calculated with ease. Regarding the output layer

(6) $$\begin{array}{c} \Delta \omega_{jk}=\eta o_{j}\left(d_{k}-o_{k}\right)o_{k}\left(1-o_{k}\right). \end{array}$$

For the hidden layer,

(7) $$\begin{array}{c} \Delta \nu_{ij}=\eta o_{j}\left(1-o_{j}\right)\overset{K-1}{\underset{k=0}{\sum }}\delta_{k}\omega_{jk}o_{i}. \end{array}$$

The magnitude of each component value is somewhat varied because the input is the students' grade based on the percentage system, so it needs to be normalized. The maximum-minimum method is used in this study because it processes data in a linear manner, which helps better preserve its original meaning and prevent information loss. The equation reads as follows:

(8) $$\begin{array}{c} X=\frac{I-I_{\min}}{I_{\max}-I_{\min}}. \end{array}$$

In the formula, *X* is the normalized NN input value; *I* is the unprocessed NN input value; and *I*_max_ is the minimum value of the NN input. The kind of output data affects how many neuron nodes there are in the output layer. The instructional assessment result is employed as the output variable of BPNN because the instructional assessment prediction model predicts the instructional assessment of teachers. If the output layer neuron's anticipated output vector is

(9) $$\begin{array}{c} T_{S}=\left[T_{1},T_{2},T_{3},\cdots ,T_{N3}\right]. \end{array}$$

The actual output vector is

(10) $$\begin{array}{c} O_{S}=\left[O_{1},O_{2},O_{3},\cdots ,O_{N3}\right]. \end{array}$$

Then, the correction error of each neuron in the output layer is

(11) $$\begin{array}{c} d_{s}^{k}=\left(t_{s}^{k}-o_{s}^{k}\right)o_{s}^{k}\left(1-o_{s}^{k}\right)s=1,2,3,\cdots ,N_{3}. \end{array}$$

According to the calculated correction error *d*_*s*_^*k*^, *whs*, and *yh* of each neuron in the output layer, the correction error of each neuron in the hidden layer can be calculated as

(12) $$\begin{array}{c} e_{h}^{k}=\left[\overset{n3}{\underset{s=1}{\sum }}d_{s}^{k}w_{hs}^{k}\right]y_{h}^{k}\left(1-y_{h}^{k}\right)h=1,2,3,\cdots ,N_{2}. \end{array}$$

Choosing the right network structure is a crucial effort. A three-layer network structure is used in this paper. It is determined that NN has 23 nodes in its input layer. The output layer of the network is only configured with one output node because there is only one instructional level assessment result. Preprocessing should be done on the data before training the NN algorithm. The performance and outcomes of the assessment algorithm will be directly impacted by the preprocessing quality of the original teaching-related data. In this study, the data normalization approach is used, and all the data are processed using a linear transformation in the (0, 1) or (-1,) range. To allow for the naturalization of all assessment indices in the range (0, 1), the actual data sample value is divided by the index's ideal maximum value. Each instructional level assessment index employed in this study is used to create the input vector for a NN. The evaluation value or the outcome of experts' assessments is what makes up the output vector of a NN. The necessary classroom instructional level assessment model is the network model obtained up until the system fault satisfies the stipulated requirements. This study also uses a modified gradient descent approach to quicken network learning's rate of convergence.

## 4. Result Analysis and Discussion

MATLAB is a commercial mathematics software, which contains an NN toolbox. This toolbox mainly aims at the analysis and design of NN system, and provides a large number of functions, graphical user interfaces and Simulink simulation tools that can be called directly. It is one of the excellent software for the analysis and design of NN system. MATLAB can save a lot of programming time. In this paper, the NN toolbox in MATLAB is used to simulate the feasibility of NN model for instructional level assessment. The training situation of the network is shown in Figure 3.

The sample selection should choose representative classrooms based on summary and analysis, develop classroom instructional questionnaires in accordance with instructional level assessment indices, and then choose and grade each indice. The instructional supervision team's evaluation of each teacher's performance in the classroom is employed in this study as a technical index, and the data is used to create a data network. In this approach, the assessment findings include both the supervision team's guiding principles and the students' viewpoints. In this study, various indicator levels are chosen, and multiple methods are put to the test repeatedly. MSE (Mean Squared Error), RMSE (Root Mean Square Error), and MAE are these metrics (Mean absolute error). The experiment demonstrates that the algorithm's MSE is depicted in Figure 4.  Figure 5 displays the algorithm's RMSE.  Figure 6 displays the algorithm's MAE scenario.

The beginning weight depicts the NN training's initial position on the error surface. In this study, several small random numbers are chosen for initial weights in the network training process over a number of iterations, and the training results are compared to choose the group of random numbers with the minimum final output error.  Figure 7 displays the assessment accuracy of several algorithms.

After training, it is proved to be a reasonable NNMATLAB program, which can be further transformed into an assessment component of VC++ program. The generated assessment component can be directly copied to the specified directory of the instructional assessment system, and the packaged component can be directly applied to the teacher's instructional assessment system in this paper, and can be called by the software on the user's operation layer.

In order to reflect the experimental results more intuitively, this paper draws the results into tables.  Table 2 shows the experimental results obtained by several algorithms.

Experimental results show that the assessment accuracy of this algorithm can reach 96.11%, which is about 13% higher than that of the traditional NN method. This shows that it is completely feasible to use NN to evaluate instructional level, and it can meet the accuracy requirements. The assessment results after network training and expert assessment results are shown in Table 3.

The experimental results show that the training and prediction accuracy of the instructional level assessment model based on BPNN is completely within the acceptable range. It is a reasonable and feasible prediction model and provides a convenient and practical tool for instructional level assessment.

## 5. Conclusion

The art of communicating emotions through music makes music education a crucial component of competence education. Education in music has a priceless impact on college students' overall quality, personality development, and mental hygiene. The healthy growth of people themselves serves as the cornerstone of competence education. The education at teachers' university, notably the overall caliber of music majors there, is crucial since it is the mother of competence education. This essay conducts a thorough investigation into the evolution of college music education and the reform of music education at teachers' universities based on the notion of competency education. This essay first examines the significant contribution that music instruction makes to the development of a student's all-around character. This essay examines the current state of the music education curriculum system at teachers' university and suggests some potential reform routes. Second, this research builds an evaluation model of music instructional level based on NN algorithm to assess music instructional level. A rich fundamental data set for instructional assessment has been created on this premise through the evaluation of instructional specialists, teachers' peers, and students. The construction of a hierarchical optimization of the classroom instructional level assessment index system is also shown. It entails selecting topics for comprehensive instructional level assessments and creating a hierarchical index system for instructional level assessments based on the features of academic fields and colleges. The proposed model is then enhanced and validated, offering a workable answer for the level of teaching assessment model in music. According to experimental findings, this algorithm's evaluation accuracy can reach 96.11%, which is almost 13% greater than that of the conventional NN technique. The accuracy of this model's assessment is good, and there is little discrepancy between the output value and the actual value. This outcome demonstrates the accuracy and dependability of the model. This study is intended to serve as a reference for the advancement of collegiate music education as well as the reform and innovation of music in teacher education programs. The next stage will be to increase the level of componentization further in order to enhance the system's maintainability and scalability. It is thought that a suitable hope road for the healthy development of music education in universities can be explored as long as every music teacher fully understands that the essence of music education is a kind of creative education of great significance to cultivate college students' aesthetic ability, creative spirit, and innovative ability.

## Figures and Tables

**Figure 1:** Neuron model.

**Figure 2:** BPNN model structure.

**Figure 3:** Training of the network.

**Figure 4:** MSE situation of algorithm.

**Figure 5:** RMSE situation of algorithm.

**Figure 6:** MAE situation of algorithm.

**Figure 7:** Assessment accuracy of different algorithms.

**Table 1:** Specific content table of music instructional level assessment index system.

Primary index	Secondary index
Instructional attitude	Rigorous lesson preparation and complete lesson plan
	Correct homework and tutor students

Instructional ability	Systematization of content
	Complex problems are clearly expressed
	Integrating theory with practice
	Auxiliary instructional means
	Treatment of key and difficult points
	Language and writing on the blackboard
	Mobilize students' enthusiasm

Instructional content	Proper selection of content
	Accurate and clear concept
	Give prominence to the key points

Instructional method	Flexible method
	Pay attention to inspiration and ability.
	Pay attention to communication and interaction with students

Instructional and educating people	Teach and educate people, be a teacher by example
	Be strict and fair to students

Instructional effect	Students master all knowledge points.
	Improve students' comprehensive ability

Student assessment	Students' mutual assessment
	Supervision and assessment
	Teachers' assessment of learning
	Student self-assessment


**Table 2:** Experimental results of each index of the algorithm.

Algorithm	MSE	RMSE	MAE	Assessment accuracy
Traditional NN	0.115	0.324	0.582	0.831
Traditional genetic algorithm	0.109	0.309	0.547	0.842
*K*-means algorithm	0.095	0.287	0.578	0.865
Methods of this paper	0.071	0.245	0.523	0.961

**Table 3:** Comparison between NN training results and actual assessment results.

Algorithm	1	1	3	4	5	6
Expert assessment	0.784	0.859	0.859	0.761	0.912	0.854
Network assessment	0.790	0.862	0.866	0.754	0.916	0.857

## Data Availability

The data used to support the findings of this study are available from the corresponding author upon request.

## References

[1] Ni Z., Wang F. (2022). Quality Assessment of Vocational Education Teaching Reform Based on Deep Learning. *Computational and Mathematical Methods in Medicine*.

[2] Parkes K. A., Daniel R., West T., Gaunt H. (2015). Applied music studio teachers in higher education: exploring the impact of identification and talent on career satisfaction. *International Journal of Music Education*.

[3] Pan W. T., Huang C. E., Chiu C. L. (2016). Study on the performance assessment of online teaching using the quantile regression analysis and artificial neural network. *The Journal of Supercomputing*.

[4] Hall W. A. (2013). Consumerism and consumer complexity: implications for university teaching and teaching evaluation. *Nurse Education Today*.

[5] Shrestha S. (2018). Mathematics art music architecture education Culture. *Nexus Network Journal*.

[6] Mccabe R. B. M., Brown A. R. (2008). Computers in music education: amplifying musicality. *Computer Music Journal*.

[7] Cheng L., Wong P., Chi Y. L. (2020). Learner autonomy in music performance practices. *British Journal of Music Education*.

[8] Van der Merwe L., Habron J. (2015). A conceptual model of spirituality in music education. *Journal of Research in Music Education*.

[9] Bonastre C., Mu Oz E., Timmers R. (2017). Conceptions about teaching and learning of expressivity in music among higher education teachers and students. *British Journal of Music Education*.

[10] Tobias E. S. (2015). Crossfading music education: connections between secondary students' in- and out-of-school music experience. *International Journal of Music Education*.

[11] Hayes L. (2017). Sound, electronics, and music: a radical and hopeful experiment in early music education. *Computer Music Journal*.

[12] Conway C., Vaughan-Marra J., Marra C. (2021). Balancing the varied needs of master of music education students: perceptions from program directors and alumni. *Journal of Research in Music Education*.

[13] Sims W. L., Cassidy J. W. (2020). Impostor feelings of music education graduate students. *Journal of Research in Music Education*.

[14] Daubney A., Fautley M. (2020). Editorial research: music education in a time of pandemic. *British Journal of Music Education*.

[15] Gould J. L. (2014). Modernizing minds in El Salvador: education reform and the cold war, 1960–1980. *Journal of Latin American Studies*.

[16] Lockhart B. J., Capurso N. A., Chase I. (2017). The use of a small private online course to allow educators to share teaching resources across diverse sites: the future of psychiatric case conferences?. *Academic Psychiatry*.

[17] Hessler M., Pöpping D. M., Hollstein H. (2018). Availability of cookies during an academic course session affects evaluation of teaching. *Medical Education*.

[18] Amaele S. (2013). Quality education, the best pro-active measure to examination malpractices in our formal institutions of learning. *Frontiers in Molecular Neuroscience*.

[19] Liu Q., Louis P. C., Lu Y. Simtriplet: Simple Triplet Representation Learning with a Single Gpu.

[20] Zhao M., Liu Q., Jha A. VoxelEmbed: 3D Instance Segmentation and Tracking with Voxel Embedding Based Deep Learning.

[21] Philip T. M. (2013). Experience as college student activists. *Urban Education*.

